The article "Synthesis of SiO2 Nanoparticle Epoxy Resin Composite and Silicone-Containing Epoxy Resin for Coatings" was retracted in 2023. Reasons: signs of a paper mill; suspected computer-generated content; unreliable results or conclusions; concerns about the data.

# Synthesis of SiO_2_ Nanoparticle Epoxy Resin Composite and Silicone-Containing Epoxy Resin for Coatings

**DOI:** 10.1155/2022/8227529

**Published:** 2022-08-25

**Authors:** Shengwen Wang, Yinxiang Qiu

**Affiliations:** College of Chemical Engineering, Yangzhou Vocational and Technical College of Industry, Yangzhou 225127, China

## Abstract

Due to its unique properties, including strong adhesion force, high heat resistivity, high insulation properties, and strong mechanical properties, epoxy resin is the most commonly used material for a variety of applications, including adhesives, electronic devices for coatings, and somewhere as a matrix for reinforcement of composites as a fiber network. To boost their properties, different other materials are also inserted in their structure and made its composites; silicon is one of them. Corrosion is serious for marine equipment and causes economic loss. To overcome such issues, different types of coating materials are developed. In this review, current methods for coatings of different materials using a silicon dioxide epoxy nanocomposite are discussed in diversity with the currently followed synthetic routes for the preparation of nanosilica epoxy composites and enhanced properties.

## 1. Introduction

Prileschajew first developed epoxy resins in 1909. These resins are monomers having low molecular mass containing an epoxide group in their structure. A characteristic unit of epoxy polymer is the epoxide group, also called oxirane or ethoxyline, where *R*_1_, *R*_2_, *R*_3_, and *R*_4_ represent aryl and alkyl groups (Figure 1) [1, 2].

These resins are multifaceted crude materials for industrial goods including from windmill blades up to very complex aircraft portions such as wings and fuselages, as well as building coating and adhesions. These are also used in large quantities in different instruments like UV-cured electronic cured adhesions, microelectronics, and generator encapsulations. These are more often utilized for aerospace applications, as structural adhesives for automotive, for shipbuilding for protection from rusting, and as mentioned above for windmill blades. In response to such large applications of epoxy resin, scientists developed an enormous range of epoxy resin ranging from less viscous to dense, small-chain to large-chain aliphatic, like hexanediol diglycidyl ether (DGE) to high performance, diversified functionalized with aromatic groups resins like triglycidyl ether aminophenol and methyl aniline (TGMDA) [3]. Bisphenol A's DGE's (DGEBA) oligomers are the most commercially available resins, when this cures and produces thermosetting long-chain polymers, which reacted with hardners [4, 5]. Epoxies are of two main types, i.e., non-glycidyl and glycidyl epoxies. Glycidyl amine, ester, and ether are the synonyms of glycidyl epoxy resins. Epoxy resins are not gylcidylated [6].

The article "Synthesis of SiO2 Nanoparticle Epoxy Resin Composite and Silicone-Containing Epoxy Resin for Coatings" was retracted in 2023. Reasons: signs of a paper mill; suspected computer-generated content; unreliable results or conclusions; concerns about the data.

Being a thermosetting resin, these are cured using a different variety of chemicals in its curing process. The specific combination of epoxy resins and curing chemicals used determines their quality. Due to the versatile properties of these resins used for a variety of applications including fiber reinforcement products, some general adhesives, and coating applications, these applications are due to their strong mechanical properties and good resistivity to heat and chemical changes [7–13].

Fillers are required in several epoxy resin formulations. Fillers increase mechanical properties like rigidity, modulus, and hardness. But sometimes it has a negative impact on the viscosity of resins, making them unsuitable for a variety of applications. Furthermore, the filler is filtered out by the fabric when the resin product containing the filler is exposed to injection manufacturing techniques for fiber-reinforced composites. As a result, many activities that might be advantageous from the use of a filler are incompatible with standard *μ*m liners, and fillers cannot be used in transparent applications.

A composite is a material that has been blended from two or more components to produce something new with better qualities. Composites have attractive properties such as thermal stability, dynamic property, and tensile strength, making them very applicable in different applications. So these variations in properties make it a very useful material among all others. The components are macroscopically mixed and are not soluble in one another. The matrix phase is one of the constituents, whereas the reinforcing phase is the other [14].

The introduction of surface-modified nanosphere into the market was first time done in 2002 and 2003. They were created in situ immediately in the epoxy resin to use a modified sol-gel process, with a mean particle size of 20 nm and an exceedingly narrow particle size dispersion [3]. Odegard et al. [15] in their research showed molecular simulations of such particles with numerous hydroxyl groups on the aggregate surface. The industrially generated particles had a surface coating added to them. The hydroxyl treatments were applied with silanes to prevent aggregation and render the particles suitable for the resin. Despite this, some hydroxyl groups remained, making the particles somewhat acidic. It is crucial to keep this in mind while looking at various epoxy resin additives. Industrial material with an average size of around 20 nm is separated into spherical granules as excesses in epoxy resins, which is quite comparable to the model.

The article "Synthesis of SiO2 Nanoparticle Epoxy Resin Composite and Silicone-Containing Epoxy Resin for Coatings" was retracted in 2023. Reasons: signs of a paper mill; suspected computer-generated content; unreliable results or conclusions; concerns about the data.

They offer several benefits, including the fact that because they are 20 nm in size and completely monodisperse, they only have a little effect on resin viscosity at higher concentrations. Unlike fumed silica, they have no highly viscous properties and act like a Newtonian liquid. Because of their small size, they are transparent and can easily enter even close-meshed materials in composite fabrication [15].

As a result, epoxy resin formulators find them to be a very appealing raw material. After 10 years, they are still being used in a range of industrial applications, including enveloping resins, sealants, and composites like vehicle and machine components. They improve strength, modulus, rigidity, toughness, and scratch resistance, among other properties. When the epoxy resin was treated with nanosilica, significant increases in fatigue performance were reported. In this review, we will summarize the current synthesis of nano-SiO_2_ epoxy resin composites for coatings [3].

The expenses of corrosion and corrosion prevention are expected to account for a significant portion of the Western world's gross national product [16].Corrosion issues are plain of enormous importance in modern communities, even though the significance of such figures is usually contested. Corrosion can cause structural failures with disastrous implications for persons and the environment, in summing up to the financial expenses and technological overwaiting [17, 18]. Organic and inorganic coatings have long been used to shield metals against corrosion. The production of high-efficiency protective coatings for anticorrosive reasons in the marine and protection sectors requires deep knowledge and comprehension of the interconnections between both the components in coatings [19].

Among the materials, the environmentally friendly effect of silicon as a flame retardant makes it very crucial in material development especially as a composite part with epoxy resin in their composites. In the structure of silicon-epoxy resin, the silanol ether connection which is considered hydrolytically unstable is formed by reacting epichlorohydrin with sodium salts of di- and polysilanol. Mainly, silicon-bearing epoxy resin is produced by two methods. Firstly, a hydrosilylation reaction is performed for the introduction of siloxanes into the epoxy-containing moiety. Secondly, transesterification between glycidol and alkoxyl silane can also be made possible by condensing the hydroxyl-terminated end with the epoxy resin of epichlorohydrin, which makes the resin utilization as both, i.e., epoxy resin and silicone resins [20–23].

The article "Synthesis of SiO2 Nanoparticle Epoxy Resin Composite and Silicone-Containing Epoxy Resin for Coatings" was retracted in 2023. Reasons: signs of a paper mill; suspected computer-generated content; unreliable results or conclusions; concerns about the data.

## 2. Synthesis of Silicone-Based Epoxy Resin Composites

### 2.1. Siloxane-Epoxy Resin

Mercado et al. [22] prepared cured epoxy resins fabricated with silicone; their organic structures are shown in Figure 2. The cured epoxy resins have a moderate *T*_*g*_ and a high limited oxygen index (LOI) value.

Liu et al. prepared some new silicon-fabricated aliphatic epoxy resins for the application as electronic packing depiction in Figure 3 shows their chemical structure. The outcomes of these prepared cured epoxy resin for thermal stability and mechanical strength were found to be outstanding.

Park et al. [21] prepared DGEBA-Si, silicon consisting of epoxy resin by mixing DGEBA with dichloro diphenyl silane in the presence of triphenylphosphine as the catalyst. Experimental results showed that the prepared cured epoxy resin has lower *T*_*g*_ and high mechanical strength than the pure DGEBA epoxy resin.

Wang et al. [12] prepared with increased thermal stability, tensile strength, and high lap shear epoxy terminated silicon dioxide-containing resins and cured epoxy resin.

Bin et al. synthesized SiO_2_-epoxy composite (depicted in Figure 4) for the coatings to strengthen basalt fiber using a sol-gel method for SiO_2_ nanoparticle preparation, and modification was performed using a coupling agent which efficiently enhanced the tensile strength of basalt fibers as compared to pure epoxy resin [24].

Peng et al. is the founder of epoxy resin synthesized using nucleophilic substitution reaction. They used OH-Spiro-DFO and diphenyldichlorosilane and epichlorohydrin for the synthesis of DEPFS (diphenyl (9,9-di-(4-(2,3-epoxypropoxy) phenyl)-4,5-diazafluorenoxysilane) epoxy resin, as shown in Scheme 1. It was mixed with bisphenol A epoxy resin (E-51) to enhance the toughness and tensile strength of the thermoset blend [25].

Cheng et al. synthesized TEMPS (tri(3,4-epoxycyclohexylmethyloxy) phenyl silane) which is a tricycloaliphatic epoxy resin for UV-curable flame-retardant coating purposes. Initiation from the reduction of 3-cyclohexene-1-carboxaldehyde followed by a reaction with phenyltrimethoxyl silane in the presence of tetraisopropoxide as a catalyst, which was finally oxidized by *m*-chloroperbenzoic acid (mCPBA), is shown in Scheme 2. The synthesized silicone-modified epoxy resins were mixed with a commercial one with improved results in flame retardancy and decomposition temperature [26].

Yuan et al. prepared vinyl-containing epoxy resin prepolymers, vinyl terminated silicone oil, and hydrogen-containing silicone oil through hydrosilylation reaction for the construction of epoxy-containing silicone rubber, as shown in Scheme 3, which enhanced the tensile, adhesion, and thermal degradation of epoxy resin-modified silicone rubber.

The article "Synthesis of SiO2 Nanoparticle Epoxy Resin Composite and Silicone-Containing Epoxy Resin for Coatings" was retracted in 2023. Reasons: signs of a paper mill; suspected computer-generated content; unreliable results or conclusions; concerns about the data.

### 2.2. Nanosilica/Epoxy Resin Composites

Surface modification of fibers or nanoparticles and resin alteration increase component bonding and particle dispersion in the resin. This research involved the remodeling of epoxy coating and the surface treatment of nano-SiO_2_ particles.

Xiaohua et al. prepared nanosized silicon dioxide-incorporated cycloaliphatic epoxy resin 3,4-epoxycyclohexylmethyl-3′,4′-epoxy cyclohexane carboxylate by modifying the surface of SiO_2_ using *γ*-glycidyloxipropyltrimethoxysilane (KH-560) as a coupling agent. The resulted product showed enhanced toughness of cycloaliphatic epoxy resin including thermal stability and because of the perturbing of crack front, which causes altering the path change of craking [27].

Skachkove et al. reported the silicon dioxide and epoxy resin nanocomposite for the heat retardancy by the curing process of diepoxide 3,4-epoxycyclohexylmethyl-3,4-epoxycyclohexane carboxylate and SiO_2_ nanoparticles grafted with glycidyl group which showed high heat resistance for coating purpose which is nanoparticle content and curing agent dependent [28].

Li et al. prepared nanoparticulate impregnated SiO_2_ in epoxy resin for coating on carbon steel. The coating with 2 wt% nanoparticulate SiO_2_ had the highest corrosion resistance, which might be related to the production of a more compressed and waterproof polymer net in the coverings, which demonstrated excellent ionic resistance and a low diffusion coefficient for hostile medium inward migration [29].

Gang et al. prepared SiO_2_/epoxy composite to enhance the thermodynamic properties of epoxy resins using three different combining materials (agents) with variable side carbon length diversified nano-SiO_2_ and dope epoxy resin, 3-[2-(2-aminoethylamino)ethylamino]propyl-trimethoxysilane (TAPS), 3-[2-(2-aminoethylamino)ethylamino]propyl-trimethoxysilane (KH-550), and aminoethyl)—aminopropyltrimethoxy. Relative to an undoped nanoscale model, the surface-mounted KH792 form of nano-SiO_2_ showed the most noticeable improvement in thermal characteristics. The *T*_*g*_ was enhanced by 61 K while the storage modulus increased by 276 MPa. The mechanical characteristics of a nano-SiO_2_ surface-mounted KH-792 model were about three times greater than those of the undoped nanostructured model, and the *T*_*g*_ increased by 36.5 K and the heat transfer efficiency by 24.5%, according to simulation results [30].

Mohammad et al. reported improved thermal, nanomechanical, and abrasion resistance on mild steel substrates; epoxy formulations with 1%, 3%, and 5% SiO_2_ nanoscale were used. When compared to unaltered coatings, nanomechanical characteristics like hardness and elastic modulus improved. The coatings' heat and abrasion resistance improved as the SNP content of the coatings increased. The coatings with a 5% nanoscale concentration had the best mechanical, thermal, and abrasion qualities [31].

The article "Synthesis of SiO2 Nanoparticle Epoxy Resin Composite and Silicone-Containing Epoxy Resin for Coatings" was retracted in 2023. Reasons: signs of a paper mill; suspected computer-generated content; unreliable results or conclusions; concerns about the data.

Zelinlan et al. prepared SiO_2_ epoxy resin composite for coating purposes using green chemistry, did not use any toxic chemical, and completely synthesized it in a beaker using tetraethyl orthosilicate and bis (trimethylsilyl) amine as starting material, which were used for coating purposes, showing excellent waterproof ability, mechanical stability, long-term stability, and being easily coated to any solid substrate [32].

Sironmani et al. studied corrosion and wear resistance behavior on nanosilica epoxy composite coating prepared using the sol-gel method. The thermal stability of SiO_2_ nanoparticles is superior to that of epoxy silica nanocomposites, according to TGA/DTA studies. When compared to silica microparticles, the glass transition temperature of composites was reduced. Nano-SiO_2_ combined coatings had better adhesion, wear, and scratch resistance than micro-SiO_2_ integrated coatings. Nanosilica pigmented coatings were shown to have abrasion resistance 50% higher than microsilica pigmented systems [33].

### 2.3. Nanosilica/Epoxy Composites with Other Nanoparticles

#### 2.3.1. Synthesis through the Sol-Gel Method

Yunmin et al. prepared SiO_2_ nanolayer BN via the Stober sol-gel method and further via ultrasonication prepared epoxy/SiO_2_@BN nanocomposites. Results showed that the coating thickness or filler content would decrease the enhanced effect of the strategy on thermal conduction [34].

Gazala et al. created a polypyrrole/SiO_2_ hybrid by the chemical oxidation process of pyrrole with FeCl_3_. The polymeric hybrid infused in epoxy resin was utilized in the powder coating technique to create coatings for moderate steel substrates. PCs1 (1%), PCs2 (2%), PCs3 (3%), and PCs4 (4%) are epoxy coatings generated on steel substrates, whereas PCs1 (1%), PCs 2 (2%), PCs 3 (3%), and PCs 4 (4.0%) are epoxy coatings with varying wt% loading of polymer composite (4%) [35].

Chunli et al. reported the synthesis of Fe_2_O_3_@SiO_2_ nanocomposites via a sol-gel method where Fe_2_O_3_ nanoparticles were synthesized by coprecipitation method using TEOS (tetraorthosilicate) as a SiO_2_ source, which they utilized for anticorrosion activity, showing enhanced anticorrosion activity [36].

It has also been possible to synthesize SiO_2_ “network armor” as a flame-retardant coating by hydrolyzing, condensing, and cross-linking the substrate TEOS on the surface of fibers (sol-gel method). Totolin et al. address the application of surface pressure plasma (APP) highly technological to coat biodegradable materials. The flame resistance of the modified substrate was improved. Strong ultrasonic washes did not remove the SiO_2_ networks that were connected to the substrates, suggesting that these coatings may be useful in upholstered furniture, clothes, and military applications [37].

The article "Synthesis of SiO2 Nanoparticle Epoxy Resin Composite and Silicone-Containing Epoxy Resin for Coatings" was retracted in 2023. Reasons: signs of a paper mill; suspected computer-generated content; unreliable results or conclusions; concerns about the data.

Aurelio et al. applied the “in situ” sol-gel method to prepare biobased epoxy/silica composites using TEOS and aminopropyl triethoxysilane (APTS) as a starting material. The synthesis was carried out in two steps; initially, APTS reacted with 2,5-bis[(oxyran-2-ylmethoxy)methyl] furan (BOMF) or DGEBA monomer, to produce silica nanoparticles in epoxy; in the end, both systems were cured with methyl and anhydride (MNA) [38].

#### 2.3.2. Synthesis Other Than the Sol-Gel Method

Kejing et al. described the synthesis of silicon dioxide at the exterior of graphene nanoplates to improve the reinforcement and hardness of epoxy resins. Experimental results reveal that the prepared material has high reinforcing and mechanical e5ffect as compared to that of containing fillers. The exceptional structure and restrengthening studies of graphene and silicon dioxide decreased the force concentration, which makes the propagation way more difficult and affording more load which was attributed to the chemical bond of cross-linked epoxy resins and graphene/SiO_2_ and the size of SiO_2_ depicted in figure 5 [39].

Chufan et al. produced adhesives (EP) reinforced with multiwall carbon nanotubes and nano-SiO_2_ particles (MWCNTs). The effects of nano-SiO_2_ and MWCNTs on the tensile modulus of epoxy composites as well as their strengthening processes were studied. The outcomes show that the mechanical properties of the epoxy composites have significantly improved. Composites made of nano-SiO_2_/MWCNTs/EP exhibit the finest mechanical properties. As a result of the synergistic achieving and sustaining competitive advantage of nano-SiO_2_ and MWCNTs on the EP, the degree of stress concentration can be reduced, and more energy can be absorbed. These mechanisms include the microplastic displacement effect, micropores, their divarication influence, and the knock effect of MWCNTs in the EP matrix [40].

An atomic oxygen (AO) exposure experiment was studied for nano-SiO_2_ particles which were filled with a glass fiber/polyamide composite in a ground-based atomic oxygen effect simulation facility as part of Xin's research to enhance the AO resistance feature of a spacecraft resin matrix composite. The AO resistance of this novel composite was significantly enhanced, while mass loss and erosion yield were significantly reduced. It shows that injecting these nanoparticles with resin is a good way to improve the composite's AO resistance. After a 40-hour exposure experiment, the erosion yield of glass fiber/SiO_2_/polyimide dropped to 16.4% [41].

The article "Synthesis of SiO2 Nanoparticle Epoxy Resin Composite and Silicone-Containing Epoxy Resin for Coatings" was retracted in 2023. Reasons: signs of a paper mill; suspected computer-generated content; unreliable results or conclusions; concerns about the data.

Jelena et al. developed hardener, bisphenol A DGE, and SiO_2_ nanoparticle composites that were surface diversified with the bonding agent 3-glycidyloxypropyltrimethoxysilane. The unmodified and modified nanoparticles were mixed in an epoxy resin and cured at 0.5–5 phr using a poly (oxypropylene) diamine (parts per hundred parts of resin). The nanofiller had no influence on the epoxy-amine matrix's curing process, network shape, or disintegration mechanism, but it did increase the mechanical strength of hybrid materials, particularly Young's modulus and hardness. Only 0.38% of unmodified particles remained after thermal deterioration, resulting in significantly more residue, a 30% increase in Young's modulus, and a 40% increase in the intensity, as well as improved toughness and reduced compaction creep, often without negatively impacting the reinforced material's brittleness. Increasing the fiber content resulted in a loss of several characteristics due to increased agglomeration formation [42].

Basalt flakes (BFs) have recently become popular in the maritime sector as a one-of-a-kind anticorrosion substance for preventing metal substrate corrosion in this study, BFs were changed by using 1–7 nano-SiO_2_ nanoparticles, which successfully produced a transformed BF epoxy coating. According to experimental findings, the BF epoxy resin coating modified with three nano-SiO_2_ nanoparticles had good mechanical performance, limited water infiltration (water absorption of 0.72% after 480 hours), and superior chemical toughness (surface lowering weight rate of 2.2% in alkali solution but only 1.1% in acid solution after 480 hours) (tensile strength of approximately 33.4 MPa). The attainability of employing nano-SiO_2_ microspheres to improve the chemical and mechanical characteristics of BF epoxy resin coatings is demonstrated in this work [43].

Youqing et al.'s MoS_2_ nanosheets were created to alter SiO_2_ nanoparticles to fabricate SiO_2_-MoS_2_ basic nanomaterials as well-dispersed nanofillers, which improved the corrosion protection and mechanical properties of an oil-based epoxy matrix. The findings revealed that MoS_2_ nanosheets coated SiO_2_ nanoparticles. Furthermore, MoS_2_ nanosheets might be used as a SiO_2_ reinforcing agent to strengthen the contact area between epoxy and SiO_2_ nanoparticles, thereby improving the epoxy resin's anticorrosive and mechanical qualities simultaneously, depicted in Figure 6 [44].

The article "Synthesis of SiO2 Nanoparticle Epoxy Resin Composite and Silicone-Containing Epoxy Resin for Coatings" was retracted in 2023. Reasons: signs of a paper mill; suspected computer-generated content; unreliable results or conclusions; concerns about the data.

Yapang et al. reported the preparation of SiO_2_-epoxy and SiO_2_-glass-fiber epoxy nanocomposites, using KH-560 as a coupling agent for the synthesis of nanometer-size SiO_2_ and heated with epoxy CYD-128 at 120°C to reduce the viscosity of CYD-128 epoxy, which were then homogenized and hardener agent added. The results showed that as-prepared material possesses high tensile strength, tensile modulus, and impact strength [45].

Dahao et al. studied the incorporation of the Fe_3_O_4_ and SiO_2_ nanoparticles in the epoxy-modified silicone resin an inorganic-organic hybrid of three different types of combinations such as SiO_2_ dispersion, ferromagnetic Fe_2_O_4_ dispersion, and simultaneous dispersion of both, where nanoparticles were synthesized by using the coprecipitation method. It was reported that silica has homogenously dispersed but ferromagnetic-caused agglomeration, where simultaneous addition has good dispersion of both type particles without much loss [46].

Jieyuan et al. used a eugenol-based epoxy silane-coupling agent to make nano-SiO_2_ epoxy nanocomposite in a sustainable and ecologically friendly approach.  Scheme 4 shows the hydrosilylation method used to make a eugenol-based silicone coupling agent. The researchers discovered that using a eugenol adhesive silane pairing agent with a long-chain benzene ring in the chemical composition improved silica filler suitability with epoxy resin and resulted in favorable various locations in the matrix, thereby improving the performance improvement of epoxy-cured products [47].

Harikrishnan et al. detailed how halloysite nanotubes (HNTs) were saturated using biobased epoxy resin by vacuum infiltration, and silica nanoparticles were modified with a UV activator through simple mixing to create a self-healing covering consisting of these three materials. Both were blended with pure epoxy glue made from biobased materials and then hardened [48].

Jiayao et al. found that by coating polycarbonate (PC) substrates with an acetone solution containing epoxy resin and fluorinated silica (F-SiO_2_) nanocrystals, novel superhydrophobic coatings with significant interfacial adhesion were created. Superhydrophobic F-SiO_2_/epoxy coatings adhered to the surface of PC materials with a high degree of dependability as a result of the exfoliation of PC substrates and the crystallization process caused by acetone. [49]

## 3. Coating Applications of Siloxane and Silicon Dioxide Epoxy Resin

Polysiloxane coatings have better gloss and color retention than typical organic binders, but they have inferior mechanical qualities. The increased durability compared to organic carbon-based structures can be explained in part by comparing the chemical properties of siloxane and typical organic binders. Compared to organic binders, which have a carbon-carbon adhesion of 360 kJ/mol, polysiloxane binders have a silicon-oxygen strength development of 443 kJ/mol [50].

The article "Synthesis of SiO2 Nanoparticle Epoxy Resin Composite and Silicone-Containing Epoxy Resin for Coatings" was retracted in 2023. Reasons: signs of a paper mill; suspected computer-generated content; unreliable results or conclusions; concerns about the data.

Furthermore, the siloxane coatings have already been oxidized, preventing future oxidation. Organometals or chemicals that react with the polysiloxane's side groups are commonly utilized to catalyze the curing of polysiloxane coatings. Siloxane can be chemically combined with epoxy, acrylic, or other organic compounds to create hybrid siloxane coatings, which are widely used in industry. The gloss and color retention of epoxy-modified siloxane is often better. Some writers report how adding hydroxyl-terminated polydimethylsiloxane to the DGE of bisphenol A increased its anticorrosive properties [51]. Recent research fields have been attracted by graphene oxide-based composite coatings due to their warm-like structure with improved mechanical and anticorrosion activity as well as its great strength and impermeability; graphene-based hybrid coatings have piqued researchers' interest in developing anticorrosion applications [52].

Mingdong et al. studied siloxane-based epoxy resin coating for variable temperatures, which yielded good resistance to temperatures as low as -30°C and high as 25°C for 10 days without any change, showing good resistance to mechanical changes and corrosion [53]. Similarly, Lida et al. created modified basalt flakes with varied ratios of nano-SiO_2_ microspheres, ranging from 1 to 7%. They discovered that the BF epoxy resin protective layer modified with 3% nano-SiO_2_ microspheres had exceptional chemical solidity (outer losing weight rate of 2.2% in alkali solution and only 1.1% in acid solution after 480 hours), constrained water infiltration (water absorption of 0.72% after 480 hours), and excellent mechanical effectiveness (tensile strength of approximately 33.4 MPa) [43].

Yunmin et al. studied the effect of epoxy/SiO_2_@BN composite coatings on thermal conductivity. The thermal conduction can be reduced by coating thickness and filler amount if increased. Using the fitting model for the thermal conduction suggested that the filler content increment causes an increase in thermal conductivities of boron nitride-silicon dioxide composites, and the thermal conduction increasing elements decreases [34].

Ruben et al. studied silica/siloxane epoxy resin for anticorrosion purposes. Epoxy-siloxane-silica hybrid nanomaterials with good corrosion protection and thermal and mechanical characteristics were created to act as protective coverings for metallic surfaces [54]. The reported coating by Ruhi et al.'s result shows that the prepared composites for coatings have high thermal stability and high corrosion protection efficiency of the epoxy coatings with polymer composite in 3.5% NaCl solution which was due to homogenous dispersion of SiO_2_ particles in the polypyrrole matrix [35].

The article "Synthesis of SiO2 Nanoparticle Epoxy Resin Composite and Silicone-Containing Epoxy Resin for Coatings" was retracted in 2023. Reasons: signs of a paper mill; suspected computer-generated content; unreliable results or conclusions; concerns about the data.

Zhang et al. reported Fe_2_O_3_@SiO_2_ nanocomposite to fabricate on epoxy coatings to enhance its anticorrosion performance. By verifying that the nanocomposite is homogenously dispersed and causes the increase in the anticorrosion activity of epoxy resin, Figure 7 shows the corrosion resistance mechanism [36].

ESRs modified with ferromagnetic Fe_3_O_4_ a5nd SiO_2_ nanoparticles have a soft covering for soft magnetic composites. Because ferromagnetic Fe_3_O_4_ is used, the magnetic dilution effect is reduced, resulting in improved magnetization and permeability. Inclusion of SiO_2_ in the SMCs, on the other hand, reduces Fe_3_O_4_ nanoparticle aggregation and results in higher electrical resistivity, resulting in decreased core loss and enhanced mechanical strength [46].

In literature [48], a tremendous work reported on the synthesis of a coating system that is self-healing under UV light, produced from biobased epoxy resin, halloysite nanotubes, and silica nanoparticles. A dual container autobiobased epoxy hybrid system has been developed with the potential to autonomically mend scratches and restore structural function.

Literature always led to diversification toward efficacy in productivity and perfections; one of the recent research studies was carried out on superhydrophobic epoxies, after variable studies on mechanical distortions and in various corrosive surroundings like acidic-, alkaline-, and salinity-based. The experimental results were full of outstanding ability against photooxidative and hygrothermal aging. In response, it was admired that coatings prepared for hydrophobic application have satisfaction in harsh conditions based on PC material [49]. Similarly, Assem et al. reported icephobic coating of siloxane-based epoxy nanocomposite in low temperature [55].

## 4. Conclusion

Epoxy resins being versatile raw material are utilized in a range of industrial applications which include windmill blades, particularly in complex aeronautical parts like wings and fuselages, and used as building coatings and adhesives. In the current study, we have discussed the synthesis of silicon dioxide containing epoxy resins as well as silicon dioxide epoxy composites and their application for coating as adhesives to protect precious material from being ruptured by environmental conditions, using different environmentally friendly and green approaches. Moreover, the study of its enhanced properties such as high thermal stability, with high tensile strength, high productivity, and icephobicity to self-healing coatings, was carried out.

The article "Synthesis of SiO2 Nanoparticle Epoxy Resin Composite and Silicone-Containing Epoxy Resin for Coatings" was retracted in 2023. Reasons: signs of a paper mill; suspected computer-generated content; unreliable results or conclusions; concerns about the data.

## Figures and Tables

**Figure 1:** Structural formula of the epoxy (oxirane) group.

**Figure 2:** Silicon-fabricated epoxy resin structures.

**Figure 3:** Chemical structure of silicon-containing cycloaliphatic epoxy resin.

**Figure 4:** Silicon dioxide preparation.

**Scheme 1:** Synthesis route of the DHPFS and DEPFS.

**Scheme 2:** Synthetic route of TEMPS.

**Scheme 3:** Reaction route to synthesize EKH prepolymers.

**Figure 5:** Linkage representation of epoxy resin to the hybrid material.

**Figure 6:** Synthesis mechanism of SiO_2_-MoS_2_ core-shell nanoparticles.

**Scheme 4:** Silicone-bonding agents based on eugenol preparation.

**Figure 7:** Schematic representation of the corrosion-resistant mechanisms of Fe_2_O_3_@SiO_2_/epoxy composite coatings on a metal substrate.
